The article "Two cases of Kallmann syndrome caused by a novel mutation in ANOS1: A case report" was published in 2025. Journal: Medicine (Baltimore).

# Two cases of Kallmann syndrome caused by a novel mutation in *ANOS1*: A case report

**DOI:** 10.1097/MD.0000000000042139

**Published:** 2025-04-18

**Authors:** Jin-Ke Xiong, Sheng-ke Tu, Min Shi, Kui Song, Min Li

**Affiliations:** a Department of Pediatrics, The First Affiliated Hospital of Jishou University, Jishou, Hunan Province, China; b Department of Hematology, The First Affiliated Hospital of Jishou University, Jishou, Hunan Province, China; c Department of Pharmacy, The First Affiliated Hospital of Jishou University, Jishou, Hunan Province, China.

**Keywords:** a novel mutation, *ANOS1*, case report, Kallmann syndrome

## Abstract

**Rationale:**

Anosmin 1 (*ANOS1*) was the first gene to be associated with Kallmann syndrome (KS). We identified 2 cases of KS caused by novel mutations in *ANOS1*, which expands the spectrum of known pathogenic mutations of this gene. We also conducted a literature review on KS pathogenesis, manifestations, and therapeutic options to aid clinicians in the early diagnosis and treatment of this condition.

**Patient concerns:**

Two male patients presented with penile hypoplasia, reduced olfactory function, and delayed puberty progression.

**Diagnoses:**

Both patients exhibited olfactory dysfunction, and one presented with bilateral hand movements. Both also had low levels of luteinizing hormone (LH), follicle-stimulating hormone (FSH), and androgens. Magnetic resonance imaging revealed small pituitary volumes, thin pituitary stalks, and small olfactory bulbs and tracts. Whole-exome sequencing revealed an *ANOS1* c.90_100dupTGCTGCGCGGC (p.Arg34Leufs*25) variant in both patients. Gonadotropin-releasing hormone (GnRH) stimulation tests were performed, leading to the diagnosis of KS in both patients.

**Interventions:**

Both patients received pulsatile GnRH pump therapy.

**Outcomes:**

After pulsatile GnRH pump therapy, LH, FSH, and testosterone levels, as well as penile lengths and testicular volumes, increased significantly in both patients.

**Lessons:**

This is the first report of 2 cases of KS caused by a new mutation at the *ANOS1* locus, expanding the mutation spectrum of *ANOS1* and providing data on the clinical and genetic phenotypes of KS, which will assist clinicians in the early diagnosis and treatment of KS.

## 1. Introduction

Kallmann syndrome (KS) is a type of idiopathic hypogonadotropic hypogonadism (IHH) characterized primarily by a deficiency or dysfunction in the secretion or action of gonadotropin-releasing hormone (GnRH), leading to gonadal insufficiency accompanied by hyposmia or anosmia, as well as other nonreproductive system manifestations.^[1]^ The overall incidence rate of KS is extremely low, with the lowest estimated incidence of 1 in 48,000 (1 in 30,000 for males vs 1 in 125,000 for females).^[2]^ KS is a rare genetic disorder characterized by significant genetic and clinical heterogeneity. Approximately 20 pathogenic genes associated with KS onset have been identified, among which anosmin 1 (*ANOS1*, formerly known as *KAL1*) was the first. Here, we report 2 cases of KS caused by the same, novel mutation in *ANOS1*.

The article "Two cases of Kallmann syndrome caused by a novel mutation in ANOS1: A case report" was published in 2025. Journal: Medicine (Baltimore).

## 2. Case presentations

### 2.1. Patient 1

A male 16-year-old patient was admitted to our hospital because of a small penis for 16 years. During growth and development, the patient showed no penis development, no voice change, and no Adam apple, as well as had no axillary hair and only short pubic hair growth. In addition, the patient also reported a reduced sense of smell and attenuated response to irritating odors. The patient’s height and weight increased continuously, and the vital signs were normal upon admission. The testicular volume was 3 mL, the penis was stretched to 4 cm, and the pubic hair was Tanner Stage III. The patient was 180 cm tall and weighed 87 kg, with a body mass index of 26.85 kg/m^2^. General examinations, including routine blood tests, liver and kidney function tests, electrolytes, homocysteine, thyroid function tests, parathyroid hormone, adrenocorticotropic hormone, cortisol rhythm, and insulin-like growth factor levels, were all normal. The dihydrotestosterone concentration was 34.48 pg/mL. The levels of 6 hormones are shown in Table 1. Chest radiography findings were normal. Ultrasonography revealed mild tricuspid regurgitation, bilateral breast gland development, slightly enlarged left axillary lymph nodes, fatty liver, and no abnormalities in the urinary system or prostate. The left and right testicles were small, measuring 11.9 × 8.4 mm and 12.5 × 6.9 mm, respectively. Magnetic resonance imaging (MRI) revealed small pituitary volume (height approximately 2.3 mm), poor display, and small bilateral olfactory bulbs volume (maximum right olfactory bulb width was ~1.2 mm). A nasopharyngeal cyst, suspected to be a Tornwaldt cyst, was also observed.

**Table 1:** Levels of 6 hormones measured in 2 patients with Kallmann syndrome.

Hormones	Patient 1	Patient 2	Units of measure
Luteinizing hormone	0.17	0.05	IU/L
Follicle-stimulating hormone	0.26	0.77	IU/L
Prolactin	4.93	6.60	ng/ML
Estradiol	43.59	90.28	pmol/L
Progesterone	0.25	1.39	nmol/L
Testosterone	1.32	0.49	nmol/L

### 2.2. Patient 2

A male 19-year-old patient was admitted because of a small penis for 19 years. The patient’s mother had noticed that his penis was smaller than those of the patient’s peers immediately after birth. During growth and development, the patient showed no significant penis development, no voice change, no Adam apple, and no axillary and pubic hair growth. The patient had a reduced sense of smell and responded only to irritating odors. In addition, the patient exhibited occasional bilateral hand movements. The patient’s height and weight continuously increased. The vital signs were normal upon admission. The testicular volume was 4 mL, the penis was stretched to 4 cm, and the pubic hair was Tanner stage II. The patient was 180 cm tall and weighed 84 kg, with a body mass index of 25.93 kg/m^2^. General examinations including routine blood tests, liver and kidney function tests, electrolytes, homocysteine, thyroid function tests, parathyroid hormone, adrenocorticotropic hormone, cortisol rhythm, and insulin-like growth factor 1 levels, were all normal. The dihydrotestosterone concentration was 61.57 pg/mL. The concentrations of 6 hormones are shown in Table 1. Chest radiographs showed normal findings. The ultrasonography findings revealed mild tricuspid regurgitation. Bilateral breast gland development was noted along with fatty liver, and no significant abnormalities in the urinary system or prostate were observed. The left and right testicles were small, measuring 11 × 8.1 mm and 13 × 7.6 mm, respectively. MRI revealed a relatively small pituitary volume (height approximately 5.6 mm), small bilateral olfactory bulbs and tracts (maximum width ~1.1 mm).

The article "Two cases of Kallmann syndrome caused by a novel mutation in ANOS1: A case report" was published in 2025. Journal: Medicine (Baltimore).

### 2.3. Diagnosis and treatment

Both patients were obese, had fatty liver disease, and showed breast development. MRI revealed small pituitary volume, thin pituitary stalk, and small bilateral olfactory bulbs and tracts. Both patients had low luteinizing hormone (LH), follicle-stimulating hormone (FSH), and testosterone levels. Patients 1 and 2 were cousins, and their mothers were sisters. They had first visited the urology department in childhood and were diagnosed with micropenis; however, no treatment was provided. In August 2022, they visited the urology department of another hospital and were administered oral testosterone undecanoate for 6 months, after which both patients’ penis and pubic hair developed.

On July 17, 2023, they visited the Peking Union Medical College Hospital for whole-exome sequencing (WES), the results of which are shown in Table 2. Both patients showed the same *ANOS1*; NM_000216.2:c.90_100dupTGCTGCGCGGC (p.Arg34Leufs*25) mutation.

**Table 2:** Whole-exome sequencing results.

	Patient 1	Patient 2
Gene	*ANOS1*	*ANOS1*
Chromosome location Transcript number nucleotide changes (amino acid changes) Genetic subregion Genotype Pathogenicity classification (associated diseases/patterns of inheritance)	chrX:8699977-8699978 NM_000216.2:c.90_100dupTGCTGCGCGGC (p.Arg34Leufs*25) *EX1/CDS1* semi-cohesive suspected to be pathogenic Hypogonadotropic Hypogonadotropic hypogonadism type 1 with or without loss of smell (Kallmann syndrome type 1) (OMIM:308700)/XL	chrX:8699977-8699978 NM_000216.2:c.90_100dupTGCTGCGCGGC (p.Arg34Leufs*25) *EX1/CDS1* semi-cohesive suspected to be pathogenic Hypogonadotropic Hypogonadotropic hypogonadism type 1 with or without loss of smell (Kallman syndrome type) (OMIM:308700)/XL

Both patients underwent GnRH stimulation tests, the results of which are shown in Table 3. Based on the above-mentioned symptoms, signs, and examination findings, both patients were diagnosed with KS and started GnRH pulsatile pump replacement therapy (10 µg of gonadorelin subcutaneously every 90 minutes) on September 7, 2023. The patients showed significant increases in LH, FSH (Fig. 1A and B), testosterone (Fig. 1C and D), penile length, and testicular volume on color Doppler ultrasound.

The article "Two cases of Kallmann syndrome caused by a novel mutation in ANOS1: A case report" was published in 2025. Journal: Medicine (Baltimore).

**Table 3:** GNRH stimulation test results.

Patient 1			
Hormone	Preexcitation	60 min after excitation	Unit of measure
Luteinizing hormone	0.19	0.20	mIU/mL
Follicle-stimulating hormone	1.44	1.76	mIU/mL

Patient 2			
Hormone	preexcitation	60 min after excitation	Unit of measure
Luteinizing hormone	0.05	0.20	mIU/mL
Follicle-stimulating hormone	0.82	1.46	mIU/mL

**Figure 1.** Gonadotropin levels, androgen levels, and testicular volume before and after pulsatile GnRH pump treatment. (A and B) Luteinizing hormone and follicle-stimulating hormone levels in patients 1 and 2, respectively, before and after GnRH pump pulsatile treatment. (C and D) Testosterone levels in patients 1 and 2, respectively, before and after GnRH pump pulsatile treatment. FSH = follicle-stimulating hormone, GnRH = gonadotropin-releasing hormone, LH = Luteinizing hormone.

## 3. Discussion

KS pathogenesis involves a reduced or completely absent ability of GnRH neurons in the hypothalamus to synthesize and secrete GnRH. Human reproductive functions are primarily controlled by these GnRH neurons. During embryonic development, neural crest and ectodermal cells mix in the bromine plate to produce GnRH and olfactory neurons.^[3]^ These neurons pass through the sieve plate, enter the developing olfactory bulb, and finally reach the hypothalamus via the forebrain.^[4]^ Mutations in genes that disrupt GnRH neuron development and migration can lead to KS. Pathogenic variants of ~20 genes have been clearly associated with KS onset, including those in *ANOS1*, NMDA receptor synaptonuclear signaling and neuronal migration factor (*NSMF*), fibroblast growth factor receptor 1, prokineticin receptor 2 (*PROK2R*), chromodomain helicase DNA binding protein 7 (*CHD7*), semaphorin 3A (*SEMA3A*), and SRY-box transcription factor 10 (*SOX10*).^[5]^ *ANOS1* (formerly known as *KAL1*), the first gene to be associated with KS, is located on the Xp22.31 chromosome and follows an X-linked recessive inheritance pattern. *ANOS1* consists of 14 exons, which encode a protein containing 680 amino acids. It includes a whey acidic protein domain, 4 fibronectin type III domains, a cysteine-rich N-terminal domain, and a histidine-rich C-terminal region. Anosmin 1 is related to the targeting adhesion of neural cells and axon growth.^[6]^ Its mutations affect the migration of GnRH and olfactory bulb neurons, leading to KS.^[7]^ The dysregulation or absence of olfactory bulb axons leads to hyposmia or anosmia. Simultaneously, insufficient secretion of GnRH by GnRH neurons results in inadequate secretion of LH and FSH by the pituitary gland, which, in turn, leads to reduced androgen secretion and causes gonadal dysfunction. Both patients in this study exhibited impaired olfactory function, responded only to pungent odors, and had low LH, FSH, and androgen levels. One patient exhibited occasional bilateral coordinated movements. *ANOS1* mutations occasionally lead to conditions such as short stature, cleft lip, cleft palate, dental dysplasia, shortened metacarpals, punctate cartilage dysplasia, renal hypoplasia, intellectual disability, mirror movements, and sensorineural hearing loss.^[8]^ *ANOS1* is expressed in the basement membrane and stromal tissues. Furthermore, in addition to ANOS1 presence in multiple brain regions, such as the olfactory bulb and cerebellum, ANOS1 expression is detected during embryonic development in many other tissues, including the digestive; respiratory, urogenital, cardiovascular, skin, skeletal, and muscular systems. This strong expression in various tissues may explain the heterogeneity of clinical presentations observed in patients with KS.

The article "Two cases of Kallmann syndrome caused by a novel mutation in ANOS1: A case report" was published in 2025. Journal: Medicine (Baltimore).

### 3.1. Clinical diagnosis

Gonadal dysfunction and reduced or lost sense of smell are the most typical features of KS. Fluctuations in the activity of the hypothalamic-pituitary-gonadal axis provide a good time window for KS diagnosis. Based on the involvement of GnRH in different stages of human growth and development, the symptoms of KS can be categorized according to the neonatal and childhood periods, puberty, and adulthood. GnRH neurons are active and secrete GnRH during the neonatal period; their activity stops during childhood and resumes in puberty.^[9]^ The reproductive cascade is temporarily active during the first 6 months of life, known as “mini puberty.” During this time, serum testosterone levels increase in male infants, whereas FSH and LH levels increase in both male and female infants. The increases in infants with IHH are very low. During mini-puberty in male infants, the surge in GnRH secretion creates the hormonal environment necessary for regulating the descent of the testes into the scrotum.^[10]^ Testicular interstitial cell-derived factors, including testosterone and insulin-like peptides, regulate the inguinal-scrotal phase of this testicular descent and the final anchoring in the scrotal position. Simultaneously, with the proliferation of supporting cells and seminiferous tubules, serum inhibin B and anti-Müllerian hormone levels rise sharply, typically peaking between 2 and 3 months after birth. Defects in mini puberty can lead to micropenises and cryptorchidism (undescended testicles). Therefore, this period is the time window for the early diagnosis of KS in males. No specific clinical signs are observed in female infants during this stage. The common symptoms in male adolescents include a lack of or low levels of masculinization, sexual dysfunction, and absence, whereas delayed breast development and primary amenorrhea are the most common complaints in female adolescents. The diagnosis of KS in adulthood is mainly associated with infertility and sometimes with the early onset of osteoporotic fractures.^[11]^

### 3.2. Genetic diagnosis

The application of new technologies such as WES has significantly increased the molecular diagnostic rate of patients with IHH. The coding gene exons account for only approximately 1% of the human genome, approximately 30 Mb, containing approximately 180,000 exons. However, most diseases (approximately 85%) are caused by low-frequency or rare mutations in coding genes. Additionally, WES easily achieves > 100 × sequencing depth, making it an efficient means of discovering information related to human diseases, especially in hereditary diseases such as KS. The detection rate of *ANOS1* mutations in KS is 10.3%, with approximately 160 variants identified, most of which are loss-of-function (frameshift, nonsense, and splice site).^[12]^ WES of samples from the 2 patients in the present report revealed that both had the same *ANOS1* mutation, c.90_100dupTGGCGCGGC (p.Arg34Leufs*25). The duplication of nucleotides TGCTGCGCGGC from positions 90 to 100 led to a frameshift mutation starting from the 34th amino acid, arginine (Arg), resulting in a change to leucine and incorrect encoding of the subsequent 25 amino acids. According to American College of Medical Genetics guidelines, this mutation is classified as a variant of uncertain significance, meeting the PVS1 + PM2 criteria, defined as follows. PVS1: when the pathogenic mechanism of a disease is loss-of-function, the detected variant is a nonfunctional variant (nonsense mutation, frameshift mutation, classic ± one or 2 splice mutations, start codon mutations, single or multiple exon deletions). PM2: variants not found in normal control populations in the exome sequencing project, 1000 genomes, or exome aggregation consortium databases (or extremely low-frequency sites for recessive diseases). No pathogenic or likely pathogenic incidental findings were detected in patients 1 or 2 (secondary finding _Var database). This *ANOS1* mutation has not been previously described.

The article "Two cases of Kallmann syndrome caused by a novel mutation in ANOS1: A case report" was published in 2025. Journal: Medicine (Baltimore).

### 3.3. Treatment

For patients who need to maintain secondary sexual characteristics, hormone replacement therapy is primarily used, whereas for those with spermatogenic needs, gonadotropins and pulsatile GnRH pump therapy are the primary treatments. A meta-analysis indicated that compared to the effects of the traditional testosterone therapy, gonadotropin therapy can induce puberty in adolescents and young men with IHH by improving testicular development and sperm production outcomes. The combination treatment with human chorionic gonadotropin (hCG) and FSH may significantly increase testicular volume and sperm production rates, achieving greater effects than those seen after hCG treatment alone. In terms of treatment safety, adverse reactions include acne, gynecomastia, redness, and pain at the injection sites. Pulsatile GnRH pump therapy activates the hypothalamic-pituitary-gonadal axis, induces puberty onset, and promotes gonadal maturation and gametogenesis. After receiving pulsatile GnRH pump therapy, the testicular volume, length, circumference, as well as LH, FSH, and testosterone levels in patients with KS significantly improve, and inhibin B levels also increase to some extent.^[13]^ In terms of safety, no other significant adverse reactions such as injection site redness, acne, or gynecomastia are observed, except for mild local injection site pain in a small number of patients. Among the current treatment options for KS, pulsatile GnRH pump and gonadotropin therapies rather than simple testosterone or estrogen-progestin replacement therapies are more suitable for patients with fertility needs.^[14]^ The blood-testis barrier fails to form effectively in mice with insufficient GnRH production, indicating the key role of GnRH in the formation of normal testicular structure.^[15]^ Therefore, early intervention with GnRH in patients with IHH can help establishing the blood-testis barrier before puberty, thereby increasing the chances of normal spermatogenesis and fertility. For the ultimate effect of treatment, a smaller initial testicular volume or cryptorchidism at the start of treatment is associated with a smaller final testicular volume.^[16]^ A period of FSH pretreatment before hCG + FSH or GnRH pump treatment to increase the number of Sertoli cells may also increase the final testis volume.^[17]^ In addition, the degree of olfactory dysfunction may also be related to the final testicular volume and spermatogenesis.

The article "Two cases of Kallmann syndrome caused by a novel mutation in ANOS1: A case report" was published in 2025. Journal: Medicine (Baltimore).

## 4. Conclusion

In conclusion, we report for the first time 2 cases of KS caused by a novel mutation in *ANOS1*. Our observations expands the spectrum of known *ANOS1* mutations and provides a basis for the clinical and molecular diagnosis of KS. The presence of small penises and testes with olfactory dysfunction may indicate KS. KS diagnosis has an obvious timing window, and the manifestations and windows differ according to sex. Clinicians should consider early diagnosis and appropriate interventions. Early treatment with a pulsed GnRH pump can improve pubertal growth retardation and increase the chances of normal spermatogenesis and fertility.

## Author contributions

**Data curation:** Jin-Ke Xiong.

**Funding acquisition:** Kui Song, Min Li.

**Methodology:** Jin-Ke Xiong, Sheng-ke Tu, Min Shi, Kui Song, Min Li.

**Project administration:** Kui Song, Min Li.

**Resources:** Kui Song, Min Li.

**Software:** Kui Song, Min Li.

**Supervision:** Kui Song, Min Li.

**Validation:** Jin-Ke Xiong.

**Visualization:** Jin-Ke Xiong, Sheng-ke Tu, Min Shi, Kui Song, Min Li.

**Writing – original draft:** Jin-Ke Xiong, Sheng-ke Tu, Min Shi, Kui Song, Min Li.

**Writing – review & editing:** Jin-Ke Xiong, Sheng-ke Tu, Min Shi, Kui Song, Min Li.

## References

[1] DodéCHardelinJP. Kallmann syndrome. Eur J Hum Genet. 2009;17:139–46.18985070 10.1038/ejhg.2008.206PMC2986064

[2] LaitinenEMVaaralahtiKTommiskaJ. Incidence, phenotypic features and molecular genetics of Kallmann syndrome in Finland. Orphanet J Rare Dis. 2011;6:41.21682876 10.1186/1750-1172-6-41PMC3143089

[3] ForniPETaylor-BurdsCMelvinVSWilliamsTWrayS. Neural crest and ectodermal cells intermix in the nasal placode to give rise to GnRH-1 neurons, sensory neurons, and olfactory ensheathing cells. J Neurosci. 2011;31:6915–27.21543621 10.1523/JNEUROSCI.6087-10.2011PMC3101109

[4] WraySGrantPGainerH. Evidence that cells expressing luteinizing hormone-releasing hormone mRNA in the mouse are derived from progenitor cells in the olfactory placode. Proc Natl Acad Sci U S A. 1989;86:8132–6.2682637 10.1073/pnas.86.20.8132PMC298229

[5] StamouMIGeorgopoulosNA. Kallmann syndrome: phenotype and genotype of hypogonadotropic hypogonadism. Metabolism. 2018;86:124–34.29108899 10.1016/j.metabol.2017.10.012PMC5934335

The article "Two cases of Kallmann syndrome caused by a novel mutation in ANOS1: A case report" was published in 2025. Journal: Medicine (Baltimore).

[6] FrancoBGuioliSPragliolaA. A gene deleted in Kallmann’s syndrome shares homology with neural cell adhesion and axonal path-finding molecules. Nature. 1991;353:529–36.1922361 10.1038/353529a0

[7] Díaz-BalzacCALázaro-PeñaMIRamos-OrtizGABülowHE. The adhesion molecule KAL-1/anosmin-1 regulates neurite branching through a SAX-7/L1CAM–EGL-15/FGFR receptor complex. Cell Rep. 2015;11:1377–84.26004184 10.1016/j.celrep.2015.04.057PMC4464948

[8] CariboniABalasubramanianR. Kallmann syndrome and idiopathic hypogonadotropic hypogonadism: the role of semaphorin signaling on GnRH neurons. Handb Clin Neurol. 2021;182:307–15.34266601 10.1016/B978-0-12-819973-2.00022-8PMC9039773

[9] AnderssonAMToppariJHaavistoAM. Longitudinal reproductive hormone profiles in infants: peak of inhibin B levels in infant boys exceeds levels in adult men. J Clin Endocrinol Metab. 1998;83:675–81.9467591 10.1210/jcem.83.2.4603

[10] DwyerAAJayasenaCNQuintonR. Congenital hypogonadotropic hypogonadism: implications of absent mini-puberty. Minerva Endocrinol. 2016;41:188–95.27213784

[11] BoehmUBoulouxPMDattaniMT. Expert consensus document: European consensus statement on congenital hypogonadotropic hypogonadism – pathogenesis, diagnosis and treatment. Nat Rev Endocrinol. 2015;11:547–64.26194704 10.1038/nrendo.2015.112

[12] ZengWLiJWangXJiangFMenM. ANOS1 variants in a large cohort of Chinese patients with congenital hypogonadotropic hypogonadism. Zhong Nan Da Xue Xue Bao Yi Xue Ban. 2022;47:847–57.36039580 10.11817/j.issn.1672-7347.2022.220071PMC10930292

[13] GongCLiuYQinMWuDWangX. Pulsatile GnRH is superior to hCG in therapeutic efficacy in adolescent boys with hypogonadotropic hypogonadodism. J Clin Endocrinol Metab. 2015;100:2793–9.25978110 10.1210/jc.2015-1343

[14] NordenströmAAhmedSFvan den AkkerE. Pubertal induction and transition to adult sex hormone replacement in patients with congenital pituitary or gonadal reproductive hormone deficiency: an Endo-ERN clinical practice guideline. Eur J Endocrinol. 2022;186:G9–G49.35353710 10.1530/EJE-22-0073PMC9066594

[15] WillemsABatlouniSREsnalA. Selective ablation of the androgen receptor in mouse sertoli cells affects sertoli cell maturation, barrier formation and cytoskeletal development. PLoS One. 2010;5:e14168.21152390 10.1371/journal.pone.0014168PMC2994754

[16] AlexanderECFaruqiDFarquharR. Gonadotropins for pubertal induction in males with hypogonadotropic hypogonadism: systematic review and meta-analysis. Eur J Endocrinol. 2024;190:S1–S11.38128110 10.1093/ejendo/lvad166PMC10773669

[17] DwyerAASykiotisGPHayesFJ. Trial of recombinant follicle-stimulating hormone pretreatment for GnRH-induced fertility in patients with congenital hypogonadotropic hypogonadism. J Clin Endocrinol Metab. 2013;98:E1790–5.24037890 10.1210/jc.2013-2518PMC3816270

